# Screening and Identification of Key Biomarkers in Lower Grade Glioma via Bioinformatical Analysis

**DOI:** 10.1155/2022/6959237

**Published:** 2022-01-07

**Authors:** Fangzhou Guo, Jun Yan, Guoyuan Ling, Hainan Chen, Qianrong Huang, Junbo Mu, Ligen Mo

**Affiliations:** Department of Neurosurgery, Affiliated Tumor Hospital of Guangxi Medical University, Nanning, Guangxi, China

## Abstract

Lower-grade glioma (LGG) is a common type of central nervous system tumor. Due to its complicated pathogenesis, the choice and timing of adjuvant therapy after tumor treatment are controversial. This study explored and identified potential therapeutic targets for lower-grade. The bioinformatics method was employed to identify potential biomarkers and LGG molecular mechanisms. Firstly, we selected and downloaded GSE15824, GSE50161, and GSE86574 from the GEO database, which included 40 LGG tissue and 28 normal brain tissue samples. GEO and VENN software identified of 206 codifference expressed genes (DEGs). Secondly, we applied the DAVID online software to investigate the DEG biological function and KEGG pathway enrichment, as well as to build the protein interaction visualization network through Cytoscape and STRING website. Then, the MCODE plug is used in the analysis of 22 core genes. Thirdly, the 22 core genes were analyzed with UNCLA software, of which 18 genes were associated with a worse prognosis. Fourthly, GEPIA was used to analyze the 18 selected genes, and 14 genes were found to be a significantly different expression between LGGs and normal brain tumor samples. Fifthly, hierarchical gene clustering was used to examine the 14 important gene expression differences in different histologies, as well as analysis of the KEGG pathway. Five of these genes were shown to be abundant in the natural killer cell-mediated cytokines (NKCC) and phagosome pathways. The five key genes that may be affected by the immune microenvironment play a crucial role in LGG development.

## 1. Introduction

Gliomas of the nervous system are the most prevalent primary neuroepithelial neoplasms [1, 2]. The 2016 version of the WHO classification of the central nervous system tumors states that grade I and grade II belong to lower-grade gliomas (LGGs). The LGGs occur more frequently in adults, which mainly include astrocytoma, oligodendroglioma, and oligoastrocytoma [3]. LGGs mostly happen in the age group of 30 to 45 years old, with a significant difference in prognosis. The median survival is 5 to 12 years and can be extended to 20 years with effective treatment [4]. Although LGG grows relatively slowly, it has a high recurrence rate and a tendency to turn into high-grade glioma, with a high clinical disability rate and mortality. Surgical resection is an essential initial treatment for LGGs [5, 6]. Since the pathogenic molecular mechanism is unclear, the timing and efficacy of postoperative adjuvant therapies such as radiotherapy and chemotherapy remain controversial. The genetically targeted treatment, as a new method, is still being explored for its adaptability and effectiveness [7–9]. Although some biomarkers associated with disease progression have been found, we need to explore more predictive biomarkers to identify potential targets and improve therapeutic efficacy.

Gene chip technology is a fast and effective technique for detecting differentially expressed genes (DEGs) [10]. It was proven to be a reliable gene chip technology after more than a decade of development, providing an effective technology platform for storing and retrieving genes. The bioinformatics analysis is commonly used in gene screening to find DEGs and authenticate molecular biological pathways for occurrence and development of tumors. These integrated bioinformatics methods may assist in the understanding of the disease mechanisms. Microarray raw data (GSE15824, GSE50161, and GSE86574) were first selected for analysis from the gene expression omnibus (GEO) database. Then, co-DEGs of three GSEs were verified through Venn software and STRING online tool. Following that, we employed the Database for Annotation, Visualization, and Integrated Discovery (DAVID) system to find common GSE Cellular Component (CC), Biological Process (BP), Molecular Function (MF), and Kyoto Encyclopedia of Genes and Genomes (KEGG) pathways. Furthermore, we designed protein-protein interaction (PPI) networks and examined core gene amplification utilizing cell-type Molecular Complex Detection (MCODE). Besides, these core DEGs were incorporated into the UALCAN online tool to obtain meaningful survival data (*P* < 0.05).

Moreover, we identified the interaction analysis of DEG expression between LGG and normal brain samples using a gene expression profile (GEPIA) (*P* < 0.05). The 14 core DEGs were then reintroduced, and their KEGG pathway enrichment was examined using DAVID. Finally, the five DEGs (CTSS, ITGAM, ITGB2, FCER1G, and TYROBP) were significantly enriched and functional in the phagosome and natural killer cell-mediated cytotoxicity (NKCC) pathways. In conclusion, our research identifies biomarkers that are reliable for the prognosis of LGG and can be employed as potential therapeutic targets.

## 2. Method

### 2.1. Microarray Data

GEO (http://www.ncbi.nlm.nih.gov/geo) is regarded as a vast quantity of microarray data profile with publicly downloadable gene data. Using the keywords “lower grade glioma geo accession” to search on the GEO DataSets database, three gene expression datasets (GSE15824, GSE50161, GSE86574) obtained from GEO (Affymetrix GPL570 platform, Human Genome U133 Plus 2.0 Array). The three GSEs were extracted from 15 LGG and 5 normal brain samples, 15 LGG and 13 normal brain samples, and 10 LGG and 10 normal brain samples.

### 2.2. Detection of DEGs

GEO was employed to investigate the DEGs among LGG and normal brain samples. (http://www.ncbi.nlm.nih.gov/geo/geo2r) [11]. *P* value < 0.05 and logFC (fold change) > 2 were defined statistically. Subsequently, DEGs from the three datasets have been commonly integrated using the web tool Venn diagram (http://bioinformatics.psb.ugent.be/beg/tools/venn-diagrams) [12]. LogFC < 0 was considered as an upregulation of DEGs, while logFC > 0 was a downregulation *of DEGs*.

### 2.3. DEG Enrichment Analysis by GO and KEGG Pathways

The annotation system, DAVID (version 6.8) [13], was employed for the evaluation of biological data and differentially expressed proteins. KEGG is a database that is used to evaluate and annotate gene functions and biological metabolic pathways using high-throughput experimental techniques [14]. Gene Ontology (GO) annotation is a functional analysis of the gene enrichment module based on the significant enrichment of GO functions, which mainly include MF, BP, and CC [15]. A biological investigation of DEG functioning was conducted by the DAVID online database (https://david.ncifcrf.gov/). *P* < 0.05 was considered significant [13].

### 2.4. An Examination of the PPI Network and Modules

The PPI network information was obtained from DEGs via the internet database Search Tool for the Retrieval of Interacting Genes (STRING; http://string-db.org) (version 10.0) [16]. Cytoscape software (http://www.cytoscape.org) was utilized to generate the network visuals and construct the subsequent networks as network analysis and visualizing tool [17]. We build a PPI network by Cytoscape, and the MCODE application was installed for identifying the most important modules in the functional networks. The following criteria were used to select MCODE: MCODE scores ≥ 5, node score cutoff = 0.2, degree cutoff = 2, max depth = 100, and *K* − core = 2.

### 2.5. Verification and Survival Analysis of Core DEGs

UALCAN (http://ualcan.path.uab.edu/), as a convenient, efficient, and interactive online web tool, was widely applied to evaluate the survival data of LGG patients using TCGA and CPTAC databases [18]. The *P* value, hazard ratio (HR), and 95% confidence interval (CI) are depicted in the figure. GEPIA (http://gepia.cancer-pku.cn/) is an online tool for profiling tumors and expression of the normal gene in The Cancer Genome Atlas (TCGA) database and performing interactive analyses (https://portal.gdc.cancer.gov/) [19]. We were able to correlate the expression differences of important genes in LGG and normal brain samples through the GEPIA website. Besides, hierarchical clustering (HC) of core DEGs was designed via the UCSC Cancer Genomics Browser (http://genome-cancer.ucsc.edu) [20]. *P* < 0.05 was considered to be statistically significant in all tests.

## 3. Result

### 3.1. Detection of DEGs in LGGs

The current investigation includes 40 LGG and 28 normal brain samples. Using the GEO2R online tool to obtain data, we extracted 1280, 2116, and 3183 DEGs from GSE15824, GSE50161, and GSE 86574. Following that, Venn diagram software was used to evaluate and detect the common genes between the three datasets. The findings revealed that the three GES had 206 similar DEGs in LGG samples, including 20 downregulated genes (logFC < 0) and 186 genes that were upregulated (logFC > 0) as shown in Figure 1.

### 3.2. GO and KEGG Pathway Enrichment Analyses in LGGs

DAVID was used to perform functional and pathway enrichment analysis on all 206 DEGs to examine their biological classification. The findings of the examination revealed that (1) on BP, upregulation of DEGs was mainly enriched in immune response, exogenous peptide antigen presentation, and antigen processing by MHC class II, positive regulation of T cell proliferation (Table 1, Figure 2(a)), innate immune response, and downregulation of DEGs in the oxidation-reduction process (Table 2). (2) On CC, upregulation of DEGs was particularly enriched in MHC class II protein complex, extracellular region, cell surface, and integral component of plasma membrane (Table 1, Figure 2(b)) and downregulated in intracellular ribonucleoprotein complex (Table 2). (3) On MF, upregulated DEGs were significantly enriched in the MHC class II receptor activity, MHC class II protein complex binding, peptide antigen binding, and receptor binding (Table 1, Figure 2(c)) and downregulated DEGs in nucleotide-binding (Table 2). Upregulation of DEGs was particularly enriched in the phagosome, intestinal immune network for IgA production, cell adhesion molecules (CAMs), and complement and coagulation cascades, as shown in Figure 2(d), whereas no KEGG pathways were significantly enriched among downregulated DEGs (*P* < 0.05).

### 3.3. Development of the PPI Network and Module Analysis

DEGs built a PPI network through the STRING database, which was visualized using Cytoscape software (version 3.4.0) (Figure 3(a)). The network was then subjected to a module analysis using the MCODE plugin. Two key modules were derived from the PPI network, including 58 nodes and 303 edges. The larger module consists of 22 nodes and 252 edges. The 22 nodes were included as follows: CSF1R, CCR1, C1QC, CCL4, AIF1, C1QA, LCP2, FYB, TYROBP, CD300A, PTPRC, LY86, ITGB2, FCER1G, ITGA, MNDA, CD74, CYBB, MPEG1, TLR7, CTSS, and TLR1 (Figure 3(b).

### 3.4. Analysis of Core DEGs via the UALCAN and GEPIA

UALCAN was performed to collect survival data for 22 DEGs. During the analysis, 18 DEGs were found to be substantially linked with poor survival (*P* < 0.05), including AIF1, C1QC, CCR1, CCL4, CD300A, CD74, CTSS, CYBB, FYB, FCER1G, ITGAM, ITGB2, LCP2, MNDA, PTPRC, TLR1, TLR7, and TYROBP (Figure 4).

GEPIA was then used to analyze the variations in these 18 DEG expression levels between LCC and normal brain samples. The results indicated that compared with normal brain samples, 14 of these DEGs were significantly highly expressed in LGGs (*P* < 0.05), including AIF1, CCL4, CD300A, CD74, CTSS, CYBB, FCER1G, ITGAM, ITGB2, MNDA, PTPRC, TLR1, TLR7, and TYROBP (Figure 5).

## 4. Reanalysis of 14 Key DEGs

Through the analysis of UCSC, Figure 6 shows locations in the upregulation and downregulation of these 14 key DEGs in different histological and sample types of LGGs. At the same time, the possible enrichment KEGG pathway of these 14 key DEGs was analyzed by DAVID. The results showed that three DEGs (FCER1G, ITGB2, TYROBP) and three DEGs (ITGB2, CTSS, ITGAM) were significantly enriched in NKCC and phagosome pathways, respectively (Table 3 and Figure 7).

## 5. Discussion

With the development of the molecular mechanism of LGGs, some key genes have been discovered. They can influence the formation and progression of tumors in a variety of pathways. Chromosome 1p/19q codeletion, isocitrate dehydrogenase (IDH) mutation, and O6-methylguanine-DNA methyltransferase (MGMT) promoter methylation have been proven to predict better prognosis of LGG, so they have been routinely tested by qualified medical institutions and widely used in clinical diagnosis and treatment [9, 21–23]. To identify more helpful prognostic biomarkers in LGGs, we employed bioinformatics tools and analyzed three datasets (GSE15824, GSE50161, and GSE86574). This study included 69 LGGs and 26 normal brain tissue samples. We detected 206 often altered DEGs (*P* value < 0.05 and logFC > 2) using GEO2R and Venn tools, including 186 upregulations (logFC > 0) and 20 downregulations (logFC < 0). The investigation of GO and pathway enrichment by DAVID methods then reveals the following: (1) On BP, upregulation of DEGs is principally enriched in immune response, exogenous peptide antigen presentation, and antigen processing through MHC class II, innate immune response, and positive regulation of T cell proliferation. (2) On MF, upregulation of DEGs mainly was enriched in MHC class II receptor activity, peptide antigen binding, protein complex binding, and receptor binding. In addition, through UALCAN analysis, we found that 18 of 22 DEGs were significantly associated with poor prognosis. Of the 18 DEGs identified, 14 were highly expressed in LGGs compared to normal brain tissue through GEPIA analysis (*P* < 0.05). In the end, through DAVID's reanalysis of KEGG pathway enrichment in 15 genes, we found that three DEGs (FCER1G, ITGB2, TYROBP) and three DEGs (ITGB2, CTSS, ITGAM) were significantly enriched in NKCC and phagosome pathways, respectively, and may be used as predictive biomarkers and therapeutic target for survival improvements of LGG patients:

- *TYROBP (TYRO protein tyrosine kinase binding protein)*: TYROBP is a transmembrane signaling polypeptide. It is an important signal transduction protein for many cell surface receptors in the body. It is significant in the signal transduction of osteoclasts, macrophage dendritic cells, and microglia. Meanwhile, TYROBP is associated with natural killer (NK) cell receptors to mediate NK cell activation [24]. It also enhances trafficking and cell surface expression of NK cell receptors. Besides, the TYROBP also has the function of regulating bone marrow cell activation, mediating the activation of neutrophils and mononucleoblasts, and promoting neuronal apoptosis that occurs during brain development. It has been discovered that overexpression of TYROBP is linked with several cancers and their poor clinical outcomes [25, 26]. Yang et al. indicated that inhibition of TYROBP gene expression could lead to better prognosis in patients with renal clear cell carcinoma [27]. Kelly et al. have experimentally confirmed that the microcolloids of the IDH mutants are mainly proinflammatory. The regulatory TYROBP gene, which dominates in IDH-wild GBM, has the effect of anti-inflammatory macrophages, resulting in the poor prognosis of this type of high-level glioma [28]. Our current study also found that high expression of the TYROBP contributes to poor prognosis in LGG patients.
- *FCER1G*: as a constitutive component of the interleukin-3 receptor and high-affinity immunoglobulin E (IgE) receptor complex, it is mainly involved in selectively mediating the formation of interleukin-4 (IL4) by basophils, mediating the allergic inflammatory signaling of mast cells. Previous research has found that FCER1G mediates the activation of neutrophils and platelets, playing a key role in some hematological diseases such as leukemia and platelet-related diseases [29]. FCER1G proved to be an essential molecule in widely existing signaling pathways, participating in a large number of immune responses and cellular activities [30]. Studies have confirmed that FCER1G is an innate immune FCER1G involved in the occurrence and progression of eczema, which affects the prognosis of meningioma, renal cell carcinoma, acute myeloid leukemia, and other diseases by acting on relevant immune pathways [31–33].
- *ITGB2/ITGAM*: ITGB2 and ITGAM are two distinct *α*M*β*2 chains. ITGAM/ITGB2 participates in multiple adhesion associations between monocytes, macrophages, and granulocytes, as well as mediates the uptake of complement envelope particles and pathogens [34]. ITGB2 encodes an integrin *β* chain, which interacts with multiple distinct *α* chains to form various integrins. ITGB2 plays a critical function in tumor invasion and metastasis by interacting through its major ligand ICAM-1 (intercellular adhesion molecules) [34, 35]. Meanwhile, ITGB2 plays a critical role in tumor cytotoxic immune response by mediating cytotoxic T cell or NK cell adherence to target cells. One study discovered that ITGB2-mediated neutrophil adherence to cancer cells was linked to early metastases of liver cancer. Another study that used genome sequencing discovered that detected ITGB2 was associated with vulnerability to chronic lymphoblastic leukemia [36, 37]. Through the regulation of CD18, ITGAM plays a crucial role in tumor adhesion, spreading, and migration. Blocking this pathway can significantly reduce the microparticle-mediated metastasis of tumor cells [38].
- *CTSS*: CTSS as a protease exists commonly in human tissues and cells. The biological function is mainly to remove invariant chains from MHC II molecules. It is commonly recognized to play a crucial role in inflammatory responses and autoimmune diseases [39, 40]. Cysteine cathepsin protease is considered to be a degrading enzyme that is involved in almost all critical functional processes of lysosomes, such as autophagy, antigen presentation, protein degradation, and apoptosis. It has also been widely recognized to play a vital role in malignant cell transformation, such as adhesion changes, blood vessel invasion, extracellular matrix breakdown, and distant colonization of tumors [41, 42]. Harbeck et al.'s study found that CTSS mediated breast cancer cell penetration through the blood-brain barrier by proteolytic hydrolysis of adhesion molecules [43]. Increased CTSS expression has been linked to an increase in invasive melanoma metastasis, according to studies. Similarly, CTSS has been revealed to play a vital role in accelerating tumor development, angiogenesis, and tumor invasion in pancreatic cancer [44]. Furthermore, a considerable rise in CTSS expression has been proven to be a predictor of poor prognosis for a range of cancers, such as lung, breast, and colorectal cancers [43, 45]

According to previous research, the central nervous system is an immunologically favored site. Since rodent cells implanted into the brain can survive successfully, but the same cells are eliminated by the host's immune system when placed in the external environment of the human body, Lim et al. therefore proposed the resistant immunity characteristics of the central nervous system [46]. At the same time, the central nervous system lacks lymphatic vessels and the blood-brain barrier exists; it is difficult for lymphocytes to reach the central region. According to the traditional view, the immune system mostly in the central nervous system is inactive and unable to properly interact with the immune system throughout the body. In recent years, more and more studies have found that the central nervous system has an active and tightly regulated immune system. In 2015, Louveau et al. found that there were lymphatic ducts in the brain, so antigen-presenting cells (microglia cells) of the brain could leave the center and enter the cervical lymph nodes [47]. Besides, central inflammatory states, such as intracerebral abscess, can also indicate that brain immunogens can generate a robust immune response [46, 48]. At the same time, the growth of glioma can destroy the blood-brain barrier, which is beneficial for lymphocytes to enter and leave brain tissue. Even if the blood-brain barrier is intact, lymphocytes can also cross the blood-brain barrier through the action of chemokines [49]. At present, more and more research focuses on the immune mechanism in the tumor microenvironment and the new methods of immunotherapy [49–52]. Our study confirms that FCER1G, GENE, ITGAM, ITGB2, and CTSS are associated with tumor development and prognosis, indicating that they are operational targets for future therapeutic development. More importantly, some of them are involved in NKCC and phagosome signaling pathways that play a major role in tumor microenvironment and immune mechanisms [40, 53]. It is also worth pursuing further research on tumor immunotherapy. Although numerous studies have established that these five genes are linked to the progression of several types of tumors, a review of the existing literature reveals that these five genes are rarely found in LGGs. Therefore, the data in this study can provide reliable evidence and new directions for the study of LGGs in the future.

## 6. Conclusion

To conclude, the current study is aimed at confirming the molecular mechanism of LGG progression and investigating potential biomarkers using bioinformatics analysis. Our findings revealed 14 genes that are related to a poor prognosis in LGG patients and are differentially expressed in tumor tissue and healthy brain tissue. Five genes were found to be enriched: FCER1G, GENE, ITGAM, ITGB2, and CTSS. NKCC and phagosome signaling pathways, which influence the immunological microenvironment, are predicted to play a major role in the progression of the tumor; it also provides the feasibility of current tumor immunotherapy with evidence; at the same time, these essential genes can be used as potential targets for future research. However, more research is required to demonstrate the function of these genes.

## Figures and Tables

**Figure 1:** The Venn diagram software identified 206 common genes among the three datasets (GSE15824, GSE50161, and GSE86574). Distinct colors in the figure display different datasets. (a) In the three datasets, 186 DEGs were upregulated (logFC > 0). (b) In the three datasets, 20 DEGs were downregulated (logFC < 0).

**Figure 2:** Functional assessment for common upregulated DEGs of three datasets by DAVID: (a) top 10 BP results; (b) top 10 CC results; (c) significant MF results (*P* < 0.05); (d) significant enriched KEGG signaling pathways (*P* < 0.05).

**Figure 3:** (a) Cytoscape was used to design DEGs' PPI network. (b) PPI network with 22 nodes and 202 edges yielded the most significant module. The genes that were upregulated are labeled in red. The downregulated genes are labeled in blue.

**Figure 4:** The prognostic information of 22 selected DEGs was obtained by UALCAN tools analysis. 18 of the 22 DEGs were significantly associated with a poor survival rate (*P* < 0.05).

**Figure 5:** 18 DEGs associated with poor prognosis were analyzed through the GEPIA website. Compared with normal people, LGG patients had significant expression of 14 DEGs. ^∗^*P* < 0.05. LGG tissue is depicted in red squares and normal brain tissue in gray squares.

**Figure 6:** HC of 14 key DEGs was constructed using UCSC online web tools. The upregulated gene is labeled with red lines and the downregulated gene is labeled with blue lines. In the histological type, the purple stripe represents oligoastrocytoma, the red stripe represents oligodendroglioma, and the blue stripe represents astrocytoma. In the sample type, the blue stripe represents the primary tumor, and the red stripe represents the recurrent tumor.

**Figure 7:** DAVID was used to analyze 14 selected key genes. 14 highly expressed genes related to poor prognosis in LGG tissues were reanalyzed by KEGG pathway enrichment. Three DEGs (FCER1G, ITGB2, TYROBP) and three DEGs (ITGB2, CTSS, ITGAM) were significantly enriched in NKCC and phagosome pathways, respectively (*P* < 0.05).

**Table 1:** An investigation of the GO of upregulated genes related to LGGs.

Term	Description	Count	*P* value
GOTERM_BP			
GO:0006955	Immune response	24	4.3*E*-12
GO:0019886	Antigen processing and exogenous peptide antigen presentation via MHC class II	10	1.4*E*-7
GO:0045087	Innate immune response	18	3.6*E*-7
GO:0042102	Positive regulation of T cell proliferation	8	1.1*E*-6
GO:0019882	Antigen processing and presentation	7	1.0*E*-5
GO:0007165	Signal transduction	24	3.0*E*-4
GOTERM_CC			
GO:0042613	MHC class II protein complex	8	6.9*E*-10
GO:0005576	Extracellular region	38	1.1*E*-7
GO:0009986	Cell surface	20	5.3*E*-7
GO:0005887	Integral component of plasma membrane	31	1.1*E*-5
GO:0030658	Transport vesicle membrane	6	2.3*E*-5
GO:0030666	Endocytic vesicle membrane	7	3.0*E*-5
GOTERM_MF			
GO:0032395	MHC class II receptor activity	6	1.2*E*-7
GO:0023026	MHC class II protein complex binding	6	1.7*E*-7
GO:0042605	Peptide antigen binding	4	0.001
GO:0005102	Receptor binding	10	0.003
GO:0004872	Receptor activity	7	0.02
GO:0004252	Serine-type endopeptidase activity	7	0.03

**Table 2:** An investigation of the GO of downregulated genes related to LGGs.

Term	Description	Count	*P* value
GOTERM_BP			
GO:0055114	Oxidation-reduction process	2	0.04
GOTERM_CC			
GO:0030529	Intracellular ribonucleoprotein complex	2	0.03
GOTERM_MF			
GO:0000166	Nucleotide binding	4	0.005

**Table 3:** KEGG pathway analysis of 14 key DEGs in LGGs by DAVID.

Term	Description	Count	Genes	*P* value
KEGG_PATHWAY				
cjc04650	NKCC	3	FCER1G, ITGB2, TYROBP	0.006
cjc04145	Phagosome	3	ITGB2, CTSS, ITGAM	0.02

## Data Availability

The data used to support and demonstrate the results of this investigation are available on request from the corresponding author.
